RETRACTED

# Functionalized Ferroferric Oxide Nanomagnetic Beads for Extraction of Nucleic Acid and Its Application in Early Screening of Colorectal Cancer

**DOI:** 10.1155/2021/5230666

**Published:** 2021-11-30

**Authors:** Bing Pei, Zhenjiang Zhang, Jian Sun, xiaoYan Qi, Qian Cui, you de Yan, xiaoYan Wang, Miaomiao Yang, Chunjie Song, Lingsi Yin, Juan Wu, Zhixin Geng, Yue Bang Wang, Yi Lu

**Affiliations:** ^1^Department of Clinical Laboratory, The Affiliated Suqian First People's Hospital of Nanjing Medical University, Suqian 223800, Jiangsu, China; ^2^Department of Infectious Diseases, The Affiliated Suqian First People's Hospital of Nanjing Medical University, Suqian 223800, Jiangsu, China; ^3^Department of Gastroenterology, The Affiliated Suqian First People's Hospital of Nanjing Medical University, Suqian 223800, Jiangsu, China; ^4^Department of Neurology, The Affiliated Suqian First People's Hospital of Nanjing Medical University, Suqian 223800, Jiangsu, China

## Abstract

Early screening is an important way to reduce the incidence and mortality of colorectal cancer (CRC). Fecal DNA testing stands out among many screening methods due to its high sensitivity. However, at this stage, researchers have not found a high-efficiency method for fecal DNA extraction. To this end, this work carried out a new round of exploration. Here, this experiment synthesized a kind of nanomagnetic beads (NH_2_-SiO_2_@Fe_3_O_4_) with good stability for nucleic acid extraction. A comparative study with the centrifugal adsorption column method revealed the significant advantages of the magnetic bead method in extracting fecal DNA. The DNA extracted by the magnetic bead method is of high purity, can also achieve high-throughput tests, and is more suitable for polymerase chain reaction detection, greatly simplifying the stool DNA detection process and providing a basis for the widespread promotion of early screening.

## 1. Introduction

Colorectal cancer (CRC) has become the third most malignant tumor in the world [1–4]. Statistics in 2018 show that the incidence of CRC is about 10.2%, and the mortality rate is about 9.2%. From this point of view, the health threat CRC poses to the world's population cannot be underestimated. In the study of CRC, the surgeon summarized the clinical characteristics of the disease. Most CRCs develop from normal mucosa to colorectal adenomas, and this malignant transformation generally takes a long period of time [5–8]. In addition, studies have shown that the removal of colorectal adenoma is significant in reducing the incidence of colorectal cancer. The survival rate of patients with early diagnosed colorectal cancer in the five years after surgery is much higher than that of patients with advanced CRC [9–12]. In view of this, researchers have made more efforts in the exploration of early cancer screening methods.

RETRACTED

Because the early clinical manifestations of CRC are not obvious and difficult to detect, the past CRC screening mainly relied on the general detection of asymptomatic people or patients with a family history of colorectal cancer. In recent years, screening methods based on DNA testing have been widely promoted [13–16]. According to reports, the aggressive development of cancer is often closely related to mutations in related genes. Although gene mutations cannot directly determine the occurrence of cancer, the occurrence of cancer depends on the long-term accumulation of gene mutations. Mutations can destroy the characteristics of the protein translated from related genes, such as the three-dimensional structure and quantity, and thus lead to the loss of function. In addition, differences in location and type have different consequences for gene expression. As far as protooncogenes are concerned, they normally encode some proteins that stimulate cell proliferation. When they are mutated, protooncogenes will be transformed into oncogenes, which will overactivate stimulatory proteins and lead to excessive cell proliferation. As for tumor suppressor genes, they normally code for proteins that inhibit cell growth. Mutations will inactivate the encoded proteins and uncontrollable cell proliferation. Some studies have shown that there are multiple gene mutations in the DNA testing of CRC patients, such as KRAS, P53, DCC, MCC, APC, and PIK3CA [17–19]. In the past, the sensitivity and accuracy of detecting colorectal cancer through single-gene mutations were low, but now, the combined application of multiple gene mutations as markers has greatly improved the accuracy and specificity of detecting CRC. In addition, some scholars claim that there will be two main changes in methylation status after cancer occurs, namely, hypermethylation and hypomethylation, which will show local hypermethylation and overall hypomethylation [20–23]. These findings lay the foundation for the understanding of cancer epigenome and the development of early cancer screening or preventive treatment.

In the screening of the source of DNA at the mutation site, tissue and fecal exfoliated cells accounted for a relatively large proportion. The detection method of tissue cells is cumbersome and the operability is more complicated. The colorectal epithelial cells are renewed at a rate of about 1% per hour. Compared with other cells, they have a faster renewal rate. Therefore, the detection of exfoliated cells and their mutant genes in feces can be a noninvasive method for CRC screening and early diagnosis way [24–26].

RETRACTED

As a commonly used stool DNA extraction method in domestic and foreign laboratories, the DNA extracted by the centrifugal column method has high purity. However, due to the need for more samples and repeated centrifugation, it is highly dependent on instruments and equipment, which is not convenient for high-throughput and automatic operation, so that it is unable to screen large-scale samples [27, 28]. At this stage, the maturity of nanotechnology has begun to provide new ideas. Biological nanomagnetic beads refer to superparamagnetic microspheres with small particle size. As a new effective carrier for extracting nucleic acid, they have been rapidly popularized in China and recognized by the majority of scientific researchers. Based on the principle of adsorption between specific groups modified on the surface of magnetic nanobeads and nucleic acids, under the action of an external magnetic field, the magnetic properties of magnetic nanobeads can easily achieve directional movement and enrichment and separate nucleic acids and impurities. Different from the centrifugal column method, this method is easy to operate, can realize automation, does not need organic solvents, and does not need repeated centrifugation. At the same time, its high flux characteristics are more suitable for multisample nucleic acid extraction. In view of this, the magnetic bead method has gradually become the mainstream scheme in the industry.

Based on the above background, this project developed nanomagnetic beads (NH_2_-SiO_2_@Fe_3_O_4_) for extracting fecal DNA. The magnetic core particles of the nanomagnetic beads are Fe_3_O_4_, the outer shell layer is SiO_2_, and the functional base layer is amino (-NH_2_). The subject data show that the application of NH_2_-SiO_2_@Fe_3_O_4_ nanomagnetic beads can simplify the operation process of fecal DNA extraction, and the purity of extracted DNA meets the experimental requirements. The application of nanomagnetic beads can greatly improve the experimental flux. Therefore, NH_2_-SiO_2_@Fe_3_O_4_ biological nanomagnetic beads can effectively assist the promotion of relevant research in the field of biology and is of great significance for the popularization of fecal DNA detection in CRC early screening.

## 2. Materials and Methods

### 2.1. Materials and Instruments

Ammonium ferrous sulfate (Fe(NH_4_)_2_·(SO_4_)_2_·6H_2_O) was purchased from Wuhan Xingzhongcheng Technology Co., Ltd. (Hubei, China). Ferric chloride (FeCl_3_·6H_2_O) was purchased from Jinan Yunbaihui Biotechnology Co., Ltd. (Shandong, China). Ammonia (NH_3_·H_2_O) and ethanol (C_2_H_6_O) were purchased from Guangxi Zhechuang Chemical Co., Ltd. (Guangxi, China). Ethyl orthosilicate (C_8_H_20_O_4_Si) and toluene (C_7_H_8_) were purchased from Shanghai Cathay Chemical Co., Ltd. (Shanghai, China). 3-Aminopropyltriethoxysilane (NH_2_(CH_2_)_3_Si(OC_2_H_5_)_3_) was purchased from Jiangsu Polys Biotechnology Co., Ltd. (Jiangsu, China). Buffer SA, buffer SC, buffer SH, buffer GFA, buffer GD, elution buffer TB, magnetic bead eluate, and rinse PW were purchased from Shanghai Shangbao Biotechnology Co., Ltd. (Shanghai, China). RNase A and proteinase K solutions were purchased from Beijing Soleibao Technology Co., Ltd. (Beijing, China). The adsorption column CR2 was purchased from Hepeng Biotechnology Co., Ltd. (Shanghai, China).

RETRACTED

The magnetic frame was purchased from Nanjing Kuangshi Biotechnology Co., Ltd. (Jiangsu, China). The vortex oscillator was purchased from Beijing Yousheng United Technology Co., Ltd. (Beijing, China). The centrifuge was purchased from Alfa Laval Technology Co., Ltd. (Shanghai, China). The automatic nucleic acid extraction and purification instrument and trace ultraviolet spectrophotometer were purchased from Wuxi Biotech Biotechnology Co., Ltd. (Jiangsu, China). The qPCR analysis system was purchased from Thermo Fisher Scientific (Massachusetts, U.S.A.). The transmission electron microscope was purchased from Guangdong Jinjian Laboratory Technology Co., Ltd. (Guangdong, China).

### 2.2. Preparation of Magnetic Beads

Dissolve an appropriate amount of Fe(NH_4_)_2_·(SO_4_)_2_·6H_2_O and FeCl_3_·6H_2_O (Fe^2+^ : Fe^3+^ = 1 : 3, molar ratio) in deionized water and continue stirring for 1.5 h at 65°C. Use NH_3_·H_2_O to adjust the pH of the solution to 11. After aging for 2 h, magnetic Fe_3_O_4_ is obtained by magnetic separation. Disperse the prepared magnetic Fe_3_O_4_ into the C_2_H_6_O solution and mix it evenly. Add an equal amount of NH_3_·H_2_O with a mass fraction of 25% (the mass ratio of the magnetic Fe_3_O_4_ and ethanol ammonia water mixture is 1 : 50). Add C_8_H_20_O_4_Si dropwise to the reaction system (the mass ratio of magnetic Fe_3_O_4_ to ethyl orthosilicate is 2 : 3) and continue to stir for 18 h. After centrifugation, SiO_2_-coated magnetic Fe_3_O_4_ particles were obtained. After washing SiO_2_@Fe_3_O_4_ particles repeatedly, place them in an anhydrous C_7_H_8_ solution and place them on a magnetic stirrer. Then, add 1.0 mL of coupling agent NH_2_(CH_2_)_3_Si(OC_2_H_5_)_3_ dropwise and wait for the reaction 1 d. Obtain NH_2_-SiO_2_@Fe_3_O_4_ magnetic particles.

### 2.3. Fecal DNA Extraction Experiment

#### 2.3.1. Magnetic Bead Nucleic Acid Extraction Experiment

Use a pipette to draw 100 *µ*L, 250 *µ*L, 400 *µ*L, 500 *µ*L, and 1000 *µ*L stool samples into the centrifuge tube. Add 500 *µ*L buffer SA, 100 *µ*L buffer SC, and 0.25 g grinding beads to remove the sample. For complex components, add 10 *µ*L of RNase A solution to remove RNA residues in the stool sample. Place the centrifuge tube on a vortex shaker and mix well and then heat and lyse at 70°C for 15 min. Place the centrifuge tube in the centrifuge and centrifuge at 12,000 rpm for 1.0 min. Transfer the obtained 500 *µ*L supernatant to a new centrifuge tube. Add 200 *µ*L of buffer SH dropwise to the centrifuge tube, place it in a vortex mixer and mix well, and let it stand for 10 min at 4.0°C. Centrifuge for 3.0 min at 12,000 rpm. Transfer 400 *µ*L of the supernatant to a 96-deep well plate, add 75 *µ*L of NH_2_-SiO_2_@Fe_3_O_4_ nanomagnetic beads, and put the deep well plate into an automatic nucleic acid extraction and purification instrument for nucleic acid extraction. Add 150 *µ*L magnetic bead eluate to the DNA-containing solution, and 10 minutes later, the DNA-containing solution is obtained after removing the magnetic beads.

RETRACTED

#### 2.3.2. Nucleic Acid Extraction Experiment with the Spin Column Method

Add 500 *µ*L buffer SA, 100 *µ*L SC solution, 15 *µ*L proteinase K, and 0.25 g grinding beads to centrifuge tubes containing 100 *µ*L, 250 *µ*L, 400 *µ*L, 500 *µ*L, and 1000 *µ*L stool samples, respectively. Oscillate on the rotary instrument for 20 s, interrupt for 5 s, and repeat 3 times. Incubate in a constant temperature metal bath at 70°C for 15 min, shake twice during the incubation period, and then vortex for 15 s. Centrifuge at 12,000 rpm for 3 min to obtain the supernatant. Add 10 *µ*L of ribonuclease A solution, and let it stand for 300 s when mixing is complete to remove RNA residue. Add 200 *µ*L of SH solution, shake and mix, put it in the refrigerator, let it stand for 10 minutes, and then centrifuge again. Put an equal amount of GFA solution into the supernatant. Add the mixed solution to the adsorption column CR2 and discard the waste solution after centrifugation. Drop 500 *µ*L of GD solution to the adsorber CR2, centrifuge, and remove the waste liquid. Add 700 *µ*L of rinsing solution PW containing absolute ethanol, centrifuge, and remove the waste liquid, and repeat 2 times. After standing for 12 min, the adsorption column CR2 was transferred to a new centrifuge tube, and 50 *µ*L of elution buffer TB was dropped onto the adsorption membrane. After standing for 3 min, the solution was centrifuged to obtain a DNA-containing solution.

#### 2.3.3. Detection of DNA Yield and Purity

The DNA samples extracted by different methods were dropped onto the surface of the micro-UV spectrophotometer measuring base, and the concentration of fecal DNA obtained was measured. The absorption wavelengths of the samples at 230 nm, 260 nm, and 280 nm were compared to obtain DNA purity.

RETRACTED

#### 2.3.4. The Impact of Fecal Preservation Solution Optimization on DNA Purity

Add the stool preservation solution to the stool sample, so that the stool preservation solution is submerged in the stool sample. After storing for 2 days, the DNA of the stool sample was reextracted by the magnetic bead method, and its concentration and purity were detected. It was found that its concentration and purity were significantly reduced, making it difficult to carry out subsequent experiments. After several optimizations, the reagents and dosages of the fecal preservation solution were changed, and the fecal DNA extraction experiment was repeated.

### 2.4. Real-Time Fluorescence Quantitative PCR Amplification

Strictly follow the instructions of the qPCR instrument to amplify the obtained DNA solution and observe its UV absorption spectrum.

## 3. Results and Discussion

### 3.1. Characterization of Nanomagnetic Beads

Observe the morphological characteristics of NH_2_-SiO_2_@Fe_3_O_4_ nanomagnetic beads under a transmission electron microscope, as shown in Figure 1. The average particle size of experimentally prepared NH_2_-SiO_2_@Fe_3_O_4_ nanomagnetic beads is about 100 nm and is generally spherical. Second, the biological nanomagnetic beads prepared in the experiment are evenly dispersed and have uniform particle size.

### 3.2. The Effect of Extraction Methods on Fecal DNA Purity

This experiment has studied the difference in UV absorption of different nucleic acid extraction methods, and the results are shown in Figure 2. The data show that the UV absorption spectrum of stool DNA extracted with NH_2_-SiO_2_@Fe_3_O_4_ nanomagnetic beads has obvious peaks and valleys (Figure 2(a)), while the UV absorption spectrum of stool DNA extracted by the spin column method has no obvious peaks and valleys (Figure 2(b)).

The concentration and purity of fecal DNA extracted by different methods are shown in Figure 3. Experimental results show that the concentration of fecal DNA extracted by the spin column method is higher than that of the magnetic bead extraction method (Figure 3(a)). Nucleic acid has the highest absorption peak at a wavelength of 260 nm, while the absorption peak of protein is at a wavelength of 280 nm. It can be seen from the ratio of A_260_/A_280_ that the fecal DNA protein and phenolic impurities extracted with NH_2_-SiO_2_@Fe_3_O_4_ nanomagnetic beads are relatively high. The purity of the nucleic acid is less than that of the spin column method (Figure 3(b)). The UV absorption peak of carbohydrates is at the wavelength of 230 nm. The ratio of A_260_/A_230_ shows that there are more carbohydrates and guanidine salts in the fecal DNA solution extracted by the spin column method, while the feces obtained by the magnetic bead extraction method are contaminated by more carbohydrates and guanidine salts. DNA is purer (Figure 3(c)).

RETRACTED

After studying the influence of different stool sample volumes on DNA purity, this topic selects the most suitable stool volume as the sample and uses the magnetic bead method and centrifugation method to perform stool DNA extraction experiments. The results are shown in Figure 4. It can be seen from Figure 4(a) that the peak of the DNA solution extracted by the magnetic bead method at 260 nm is more pronounced than that of the centrifugal method. The data show that the concentration of fecal DNA extracted by the spin column method is significantly higher than that of the magnetic bead method (Figure 4(b)), and the purity of the fecal DNA extracted is about the same (Figures 4(c) and 4(d)). However, from the point of view of the operation process, the steps of the centrifugation method are more cumbersome than the magnetic bead method, requiring multiple centrifugation and higher requirements on the instrument. On the contrary, the advantages of high throughput, automation, and easy operation of the magnetic bead method cannot be ignored, and it is expected to replace the spin column method after optimization.

### 3.3. The Influence of Fecal Preservation Solution on the Amount of DNA Extracted

Add a self-prepared stool preservation solution to the stool sample, so that the stool preservation solution is submerged in the stool sample. After storing for 2 days, the DNA of the stool sample was reextracted by the magnetic bead method, and its concentration and purity were detected. It was found that its concentration and purity were significantly reduced, making it difficult to carry out subsequent experiments. After several optimizations, the reagents and dosage of the stool preservation solution were changed, and the stool DNA extraction experiment was repeated. The test results are shown in Figure 5. It can be seen from Figure 5(a) that the optimized fecal preservation solution is conducive to subsequent nucleic acid extraction experiments with nanomagnetic beads. In addition, the concentration of fecal DNA extracted by the magnetic bead method has increased (Figure 5(b)), and the content of impurities such as protein and carbohydrates has been significantly reduced (Figures 5(c) and 5(d)), allowing PCR amplification.

### 3.4. Real-Time Fluorescence Quantitative PCR Amplification Results

In this experiment, 8 extracted fecal DNA samples were selected for qPCR amplification, and the change of yield in each cycle of PCR amplification reaction was detected in real time by using the change of fluorescence signal, so as to detect and evaluate the risk of CRC. The results are shown in Figure 6. The amplification curve verified that sample A, sample B, sample C, sample F, and sample G are positive samples for CRC detection, while sample D, sample E, and sample H are negative samples. It can be seen that NH_2_-SiO_2_@Fe_3_O_4_ magnetic nanobeads have far-reaching significance in fecal DNA extraction and play a positive role in promoting the popularization of CRC early screening.

RETRACTED

### 3.5. Discussion

The popularization of early screening is a great measure for mankind to overcome the difficulties of CRC. However, the current early screening methods for CRC are still insufficient. Clinical studies have found that the detection of fecal exfoliated cell DNA can provide a lot of relevant information for CRC screening. Therefore, this study has made some efforts in the efficient extraction of fecal DNA.

In this work, ferrous ammonium sulfate and ferric chloride were used as raw materials to prepare magnetic Fe_3_O_4_ particles, and the problem of easy agglomeration and instability of Fe_3_O_4_ nanoparticles was overcome through modification experiments. The biological nanomagnetic beads were easy to separate and preserve. It showed strong practicability in the magnetic bead nucleic acid extraction method. Specifically, this work used the magnetic bead method and the spin column method to carry out fecal DNA extraction experiments and analyzed the relationship between the concentration and purity of fecal DNA and different extraction methods and different stool volumes. The results showed that the concentration and purity of fecal DNA were close to the maximum when the amount of feces used in the centrifugation method and magnetic bead method was between 400 and 500 *µ*L, and they were suitable for real-time fluorescent quantitative PCR amplification. However, the purity of the fecal DNA extracted by the magnetic bead method is significantly higher than that of the centrifugal method, and it has the advantage of simple operation [29, 30].

In conclusion, the extraction of high-quality fecal DNA is very important for related research and transformation application. In this study, the magnetic bead nucleic acid extraction method has significant advantages, which are conducive to the development of high-throughput CRC early screening.

## 4. Conclusion

The NH_2_-SiO_2_@Fe_3_O_4_ prepared in this subject has good dispersibility and stability, and its application in magnetic bead nucleic acid extraction experiments shows excellent adsorption performance. NH_2_-SiO_2_@Fe_3_O_4_ magnetic beads are easy to operate for extracting fecal DNA, with high DNA purity, and suitable for high-throughput tests. In the future, through the continuous improvement of nanomagnetic beads, magnetic bead-based nucleic acid extraction is expected to make greater contributions to the early screening of CRC.

RETRACTED

## Figures and Tables

**Figure 1:** Transmission electron microscope (TEM) image of NH_2_-SiO_2_@Fe_3_O_4_ nanomagnetic beads.

**Figure 2:** Ultraviolet absorption spectra of fecal DNA extracted by different methods. (a) Magnetic bead extraction. (b) Spin column method.

**Figure 3:** Influence of method difference on the concentration and purity of extracted nucleic acid. (a) Nucleic acid concentration. (b) Nucleic acid and protein content ratio. (c) Nucleic acid to carbohydrate content ratio.

**Figure 4:** Nucleic acid extraction experiment for optimal stool sample volume. (a) UV-Vis absorption spectrum. (b) Nucleic acid concentration. (c) Nucleic acid and protein content ratio. (d) Nucleic acid to carbohydrate content ratio.

**Figure 5:** The influence of fecal preservation solution on the amount of DNA extract. (a) UV-Vis absorption spectrum. (b) Nucleic acid concentration. (c) Nucleic acid and protein content ratio. (d) Nucleic acid to carbohydrate content ratio.

**Figure 6:** Results of qPCR amplification.

## Data Availability

The data used to support the results of this study are included within the article.
